# Raging the War Against Inflammation With Natural Products

**DOI:** 10.3389/fphar.2018.00976

**Published:** 2018-09-07

**Authors:** Ali Attiq, Juriyati Jalil, Khairana Husain, Waqas Ahmad

**Affiliations:** ^1^Drug and Herbal Research Centre, Faculty of Pharmacy, University Kebangsaan Malaysia, Kuala Lumpur, Malaysia; ^2^School of Pharmaceutical Sciences, Universiti Sains Malaysia, Gelugor, Malaysia

**Keywords:** cyclooxygenase-2, inflammation, natural products, prostaglandin E_2_, cyclooxygenase pathway, anti-inflammatory

## Abstract

Over the last few decade Non-Steroidal Anti-Inflammatory Drugs (NSAIDs) are the drugs of choice for treating numerous inflammatory diseases including rheumatoid arthritis. The NSAIDs produces anti-inflammatory activity via inhibiting cyclooxygenase enzyme, responsible for the conversation of arachidonic acid to prostaglandins. Likewise, cyclooxegenase-2 inhibitors (COX-2) selectively inhibit the COX-2 enzyme and produces significant anti-inflammatory, analgesic, and anti-pyretic activity without producing COX-1 associated gastrointestinal and renal side effects. In last two decades numerous selective COX-2 inhibitors (COXIBs) have been developed and approved for various inflammatory conditions. However, data from clinical trials have suggested that the prolong use of COX-2 inhibitors are also associated with life threatening cardiovascular side effects including ischemic heart failure and myocardial infection. In these scenario secondary metabolites from natural product offers a great hope for the development of novel anti-inflammatory compounds. Although majority of the natural product based compounds exhibit more selectively toward COX-1. However, the data suggest that slight structural modification can be helpful in developing COX-2 selective secondary metabolites with comparative efficacy and limited side effects. This review is an effort to highlight the secondary metabolites from terrestrial and marine source with significant COX-2 and COX-2 mediated PGE_2_ inhibitory activity, since it is anticipated that isolates with ability to inhibit COX-2 mediated PGE_2_ production would be useful in suppressing the inflammation and its classical sign and symptoms. Moreover, this review has highlighted the potential lead compounds including berberine, kaurenoic acid, α-cyperone, curcumin, and zedoarondiol for further development with the help of structure–activity relationship (SAR) studies and their current status.

## Introduction

Inflammation is a tightly regulated immune-protective response to combat xenobiotic invasion, mechanical, chemical, and thermal injury (Nathan, 2002; Barton, 2008). The initiation and the maintenance of the inflammation is carried out by pro-inflammatory mediators whose activity balanced out by the anti-inflammatory mediators responsible for the limiting the inflammation, once the instigating factor is removed (Segal et al., 2000; Nathan, 2002). However, there are several factors including stress (Han et al., 2002), chromosomal aberration (Shacter and Weitzman, 2002), and environmental factors (Shishodia et al., 2003) that can disturb this balance and lead to excessive production of prostaglandin E_2_, via up-regulating the COX-2 activity, which consequently leads to inflammatory mediated diseases including cancer (Pockaj et al., 2004; Misra et al., 2018), Alzheimer's diseases (Faden et al., 2016), and acute renal failure (Gomez et al., 2014; Tucker et al., 2015). NSAIDs are the drugs of choice to suppress the COX-2 associated PGE_2_ production (Ullah et al., 2016). However, the prolong use of NSAID_S_ has been associated with serious and sometimes life threatening side effects (Bjarnason and Rainsford, 2001; Mattia and Coluzzi, 2005). Hence it is imperative to find out alternative therapeutic regimen with comparative efficacy but with fewer side effects.

The natural products with medicinal properties have been used to treat all sorts of inflammatory conditions (Petrovska, 2012; Daniel, 2016). These traditional anti-inflammatory remedies later become the counter stones for the production of Aspirin, the first natural product derived synthetic anti-inflammatory drug (Attiq et al., 2017). Since then the exploration of natural bioactive compounds has been quite promising, resulting in the discovery of numinous secondary metabolites with extra ordinary bioactivities including artemisinin (Dewick, 2002), vinblastine (Cragg et al., 1997), pilocarpine etc (Patwardhan et al., 2004; Zhang L. et al., 2005). In the light of the fact, that natural products have advantageous structural diversity over synthetic compounds, makes them a potential source of novel compounds with potent anti-inflammatory activity (Tulp and Bohlin, 2002; Grabowski et al., 2008; Harvey, 2008). Henceforth this review is an effort to highlight the secondary metabolites form plant, fungi, marine and terrestrial algae source with significant COX-2 activity. Moreover, the compounds with additional PGE_2_ inhibitory activity were also included in this review, since isolates with potential to inhibit COX-2 mediated PGE_2_ production are expected to exhibit significant anti-inflammatory, antipyretic, and analgesic activity.

## Cyclooxygenase pathway

The arachadonic acid (AA) is the most essential metabolic precursor for numerous inflammatory pathways (Zeldin, 2001). It is a 20 carbon unsaturated fatty acid, widely distributed in lipid bilayer membrane in a resting position (Sevanian and Kim, 1985). However, it has been reported that numerous external and internal factor have the tenacity to activate the phospholipase A_2_ (PLA_2_). This activation cleaves the membrane bound AA from the phospholipids and makes it available for three major inflammatory pathways including cytochrome P-450 monooxygenase (Capdevila et al., 2000; De Montellano, 2005), lipoxygenase (Piomelli et al., 1987), and cyclooxygenase pathway (Kuehl and Egan, 1980; Santos et al., 2017).

The major scope of this current review is Cyclooxygenase pathway, which is considered as one of the most comprehensively studied inflammatory pathway in mammals (Shih et al., 2015). The pathway begins with the conversation of AA to PGH_2_, major metabolic substrate for the prostaglandin and thromboxane associated synthases (Sugimoto et al., 2015). This conversation take place due to the action of proton donor oxygen oxido-reductase (prostaglandin G/H synthase) commonly referred as cyclooxygenases. The whole process is carried out in two phases. In first phase, prostaglandin G_2_ (PGG2) production is carried out through oxidation of AA, which results in addition of two oxygen molecules to the AA structure (Van der Donk et al., 2002; Rouzer and Marnett, 2003). In second phase, PGG_2_ bind to the PGG_2_ specific reactive site, where the reduction of PGG_2_ take place through lipid peroxidation, which results in the production of PGH_2_ (Kawahara et al., 2015).

## Mechanism of action of cyclooxygenase pathway

The cyclooxygenase pathway initiates with the formation of hydroperoxy endoperoxide (PGG_2._) from AA (Samuelsson et al., 1978). This rate-limiting step is carried out on Carbon-13 of AA, where the abstraction of pro-S hydrogen takes place (Schneider and Brash, 2000). The activity of peroxidase is significantly important in activating and consequently making cyclooxygenase enzyme available for the reaction. Peroxide substrate undergoes two-electron reduction leading to ferric heme oxidation, which is responsible for the formation of Tyr-385, oxo-ferryl porphyrin radical-cation (Van der Donk et al., 2002). Tyr-385 reduces the heme through electron transfer and facilitates the formation of tyrosine radical at the active site of cyclooxygenase (Chandrasekharan and Simmons, 2004). This residue is important for the abstraction of pro-S hydrogen from AA which serve as a initiation signal for the cyclooxygenase reaction (Kawahara et al., 2015). In addition, the formation of PGG_2_ takes place through the reduction of peroxyl radical to the hydroperoxide (Van der Donk et al., 2002). Once activated, COX can undergo several turn over without any prior activation. Moreover, the reaction proceed with the reduction of 15-hydroperoxy of PGG_2_ to PGH_2_ (Van der Donk et al., 2002; Kawahara et al., 2015). For further clarification mechanism of action of cyclooxygenase pathway is simplified in Figure 1.

**Figure 1:** Mechanism of action of cyclooxygenase pathway.

## COX-1 and COX-2 structural and functional comparison

The cyclooxygenase enzymes can be further classified into two distinctive iso-enzymes, COX-1 and COX-2 (Fitzpatrick, 2004; Mbonye et al., 2008). COX-1 is constitutive in nature and widely expressed on various parts of the body including platelets (Crofford, 1997), kidney (Soslow et al., 2000), gastric mucosal lining (Jackson et al., 2000), duodenum (Crofford, 1997), jejunum (Crofford, 1997), and lungs (Smith et al., 2000; Chandrasekharan and Simmons, 2004). COX-1 plays significant role in carrying out numerous physiological function including platelet aggregation (Morita, 2002), hemostasis (Crofford, 1997), and protection of gastric mucosa (Brzozowski et al., 2001) and hence COX-1 is also commonly referred as “house keeping enzyme.” On the contrary, COX-2 cDNA was cloned from phorbol ester induced 3T3 fibroblasts. This discovery was a milestone in characterizing the structural and functional comparison of COX isoenzymes (Fitzpatrick, 2004). Despite its structural similarity with COX-1, enzymatic activity pattern of COX-2 is quite different due to Ptgs-2 gene. The turn over of COX-2 mRNA is relatively quicker then COX-1 mRNA due to the presence of 3′-untranslated instability sequences (Van der Donk et al., 2002; Rouzer and Marnett, 2003). Due to which COX-2 can be easily induced by various endogenous and exogenous stimulus including pro inflammatory cytokines (IL-1 and IL-6) (Samad et al., 2001), tumor necrosis factor α (TNF-α) (Wang and Smart, 1999), lipopolysaccharide (LPS) (Eliopoulos et al., 2002), and stress (Han et al., 2002; Ponik and Pavalko, 2004). Once induced COX-2 can cause excessive production of PGE_2_ (major metabolic product of COX-2) along with other prostaglandin which lower the pain threshold and induce pain, sensitize the nerve ending, increase vascular permeability and hence paving the path for inflammatory associated diseases (Mbonye et al., 2008).

The COX-1 and COX-2 consist of 576 and 581 amino acids, while both iso-enzymes share the same molecular mass of 70 kDa/monomer, along with their primary and tertiary structure (Rouzer and Marnett, 2009). Both iso-enzymes have three mannose oligosaccharides, which plays significant role in protein folding, which is responsible for imparting functional conformation to both iso-enzymes. Moreover, there is a forth-additional oligosaccharide specifically expressed on COX-2 that is responsible for the degradation and termination of its enzymatic activity. (Chandrasekharan and Simmons, 2004; Rouzer and Marnett, 2009). Structural similarly of both iso-enzymes can be judged form the fact that it has been observed that the 3D structures of both isoenzymes are almost superimposable. There are three domains present on individual subunits of dimers out of which the bulkiest one with >117 resides serve as the catalytic domain, which make up the active site for cyclooxygenase and peroxidase (Kurumbail et al., 2001; Mbonye et al., 2008). While the membrane-biding domain, which exhibit peroxidase specific active site are present on the distal part of the protein, which consist of heam group attached at the base of the cleft (Kurumbail et al., 2001). Except for the hydrophobic amino acid cluster, which makes up the dome over the cleft and repels the attachment, the rest of the structure offers high accessibility of solvent to the heam group. This structural configuration of the active site explains the COX-2 peroxidase substrate structural specificity, which limits the binding of numerous primary and secondary biosynthetic hydroperoxidase (Smith et al., 2000). Cyclooxygenase active site is present on the exterior distal part of protein which is adjacent to the L-shaped channel of the membrane-binding domain (Smith et al., 2000; Rouzer and Marnett, 2009). A specific amino acid sequence is attached at the opening of the channel. This sequence acts as a barrier, which allows the substrate and antagonist to attach with active site. Once the barrier is removed cyclooxygenase site is available for the AA binding (Rouzer and Marnett, 2009). The proceeding reaction is carried out in two phases, in phase one carboxylic group attach at the constriction, while in second phase ω-methyl gets attach to the channel terminus. Once these two attachment phases are complete, AA bends it carbon-13 into the channel allowing the attachment with Tyr-385 which initiates the cyclooxygenase reaction (Smith et al., 2000; Garavito et al., 2002).

## Role of cyclooxygenase in inflammation

COX-1 is often referred as “house keeping” enzyme due to its constitutive role in human physiology, however recent COX-1 knock out mice studies have revealed COX-1 also plays significant role in development and progression of inflammation (Langenbach et al., 1999; Kurumbail et al., 2001; Morita, 2002; Aid et al., 2008). It has been observed that COX-1 expression is up-regulated in resident inflammatory cells, responsible for carrying out acute inflammatory response and cell differentiation. In addition it has been observed that both iso-enzymes were equally expressed on adjuvant induced arthritis model and similar pattern of distribution was observed in the synovial fluid extracted from rheumatoid arthritis patients from tertiary health care centers (McAdam et al., 2000). It could be inferred from above stated studies that COX-1 associated metabolic products are associated with initiation of inflammatory acute phase, while the COX-2 expression is responsible for maintaining the inflammatory response (Schönbeck et al., 1999; McAdam et al., 2000). While the COX-2 deletion or selective inhibition in different animal models have shown ambivalent results. It has been observed that COX-2 deletion or selective inhibition may ameliorate or even worsen the inflammatory response. In few inflammatory models COX-2 deletion has caused worsening of gastric ulcers hence indicating its importance in gastric mucosal protection (Wallace et al., 2000). Likewise, in a recent study conducted to evaluate the pattern of inflammatory response in COX-1- and COX-2 knockout rat models revealed that deletion of both COX iso-enzyme can illicit acute phase inflammation. However, both models have shown variable pattern of onset, intensity and duration of inflammation. While in another study it was observed that deletion of COX-1 known gene let to the significant reversal of AA-induced edema, which exhibit significant role in resolving inflammation. Moreover, in the same study similar results were in observed where COX-2 gene deletion led to resolution of AA-induced edema in wild type COX-2 knockout model (Langenbach et al., 1995; Morham et al., 1995). Base on the above stated facts it could be inferred that both iso-enzyme play significant in early and late phase of the inflammatory response depending upon the inflammatory stimulus and degree of expression on that particular tissue (Dinchuk et al., 1995). Similarly in another study it was observed that expressions of both iso-enzyme are equally expressed in synovial fluid isolated patients suffering from synovitis. In the same study, K/BxN serum–transfer arthritis model exhibited an early up-regulation of COX-1 expression and significant increase in the production of COX-1 derived PGI_2_, which plays significant role in the development and maintenance of arthritis. While after deletion of the COX-2 in knockout model unexpectedly let to the resolution of synovial inflammation and remodeling of joint destruction (Myers L. K. et al., 2000). Moreover, in another study it was observed that COX-1 and COX-2 deletion led to the significant deceases in PGE_2_ production and reversal of inflammation in air pouch model. Additionally it was also observed that pretreatment with selective COX-2 inhibitor NS-398 (positive control) was able to resolve the inflammation and decreases the concentration of PGE_2_ in the similar manner (Langenbach et al., 1999). It was concluded from the study that COX-2 deletion have exhibited 75% fall in prostaglandin production, while COX-1 deletion in wild- type mice only led to 25% reduction in total prostaglandin production. It can be inferred from the study that both iso-ensyme are involved in prostaglandins production and COX-2 deletion may lead to resolution of acute inflammatory response (Langenbach et al., 1999). Moreover, it has been reported that cyclooxygenase iso-enzymes are likely to reverse their functional activities specifically in brain. Which is based upon an observation that intrathecal LPS administration in COX-1 knock-out mice have ameliorated the inflammatory response, while in COX-2 knock out mice inflammation was exacerbated (Langenbach et al., 1999; Smith and Langenbach, 2001; Ueno et al., 2005; Aid et al., 2008).

## Prostaglandin and inflammation

### The role of prostaglandins in mediating pain and inflammation

The PGE_2_ is responsible for maintaining numerous physiological functions including blood pressure (Armstrong et al., 1976), female reproductive system (Fortier et al., 2008), fertility (Nutting and Cammarata, 1969), protection of gastric mucosa (Lacy and Ito, 1982; Brzozowski et al., 2001), and immune response (Plescia et al., 1975; Phipps et al., 1991). However, in certain pathological conditions the level of PGE_2_ increases more than 10-fold then the normal concentration, which gives rise to serious complications. For instance, in inflammation elevated level of COX-2 mediated PGE_2_ production is responsible for exhibiting classical inflammatory sign and symptoms. PGE_2_ elevates the blood flow toward the inflamed tissue through its vasodilatory activity and increases vascular permeability (Williams and Peck, 1977). Moreover, it induces pain via sensitizing the nerve ending in both central and peripheral nervous system (Mantyh et al., 2002; Kojima et al., 2005). Furthermore, results from recent clinical trials conducted on selective COX-2 inhibitors have stated that classical NSAIDs are equally potent in reducing the PGE_2_ concentration in both isoforms (Sperling et al., 2001). Hence it can be inferred form the result that COX-2 mediated PGE_2_ production is completely dependent upon the type and site of inflammation. Moreover, recent report suggested that PGE_2_ level significant dropped after the removal of COX-2 gene form mice arthritic model and averted the overall progress of autoimmune arthritis (Myers N. et al., 2000). In recent study conducted to evaluate the PGE_2_ role in acute inflammation model suggested pretreatment with PGE_2_ monoclonal antibody and indomethacin has significant reduced that carrageenan induced edema via suppressing the COX-2 mediated PGE_2_ production (Nakatani et al., 2007). Similar results were observed in rat adjuvant arthritis rat model, where the freund's adjuvant administration leads to excessive PGE_2_ production and consequent inflammation (Mancini et al., 2001; Nakatani et al., 2007). The infiltration of monocytes and T-lymphocytes represents the inflammatory reaction, which ends up in the paw edema and joint destruction. The results suggests that the up regulation of COX-2 mRNA and COX-2 derived and PGE_2_ production was observed carrageenan induced paw edema, although no significant change was observed in COX-1 mRNA. While a significant reduction is paw volume was observed upon the administration of COX-2–specific inhibitor SC-58125, which signifies the role of COX-2 in elevated levels of PGE_2_ responsible for increase in paw volume (Guruprasad et al., 2015). Under the light of above-mentioned studies its evident that COX-2 and COX-2 mediated PGE_2_ production plays significant role in pain and inflammation.

### Microsomal prostaglandin E_2_ synthase-1 (PGES-1) and its expression

PGE synthase (PGES) is responsible for the conversation of PGH_2_ to PGE_2_. PGH_2_ is highly unstable and readily gets metabolized by COX-1 and COX-2 (Dannhardt et al., 2000; Tilley et al., 2001). So far three PGES isoforms has been reported to be involved in PGE_2_ production. PGES-1 is a membrane associated synthase and can be induced by various inflammatory mediators, while mPGES-2, and cytosolic cPGES are constitutively expressed intracellularly (Park et al., 2006). cPGES only benefits from the COX-1 activity for PGH_2_ production, mPGES-2 holds the tenacity to produce PGH_2_ utilizing both COX-isoforms (Park et al., 2006). While, inducible mPGES-1 is principally benefits form COX-2 for PGH_2_ production. mPGES-1 is a glutathione-dependent enzyme also commonly referenced as microsomal glutathione S-transferase1-like 1 (MGST1-L1) (Ricciotti and FitzGerald, 2011). mPGES-1 share inducible nature with COX-2 and both enzymes have shown patterns of synchronized induction upon receiving pro-inflammatory stimulus including TNF-α, PAF, IL-1α, and IL-6. The most significant activity of PGES is observed in COX-2 associates delayed PGE_2_ production phase. In which, pro inflammatory mediator are responsible for inducing the COX-2 dependent mPGES-1 expression (Murakami et al., 2000; Cipollone et al., 2003a). Moreover, pattern of up regulated mPGES-1 activity were also observed with hormonal stimulation, β-amyloid treatment of astrocytes. Recent studies conducted on TNF-α-induced rheumatoid arthritis synovial cells have suggested that pretreatment with dexamethasone successfully down regulated the mPGES-1 mRNA (Murakami et al., 2002). In addition it has been observed that expression of mPGES-1, PGE_2_ catalytic enzyme has seems to be unregulated in LPS-induced rat model with adjuvant arthritis. Which suggested that mPGES-1 expression can be unregulated by pro-inflammatory mediator (Tamura et al., 2016) including LPS and pro-inflammatory cytokines in various parts of the body including gingival fibroblasts, smooth muscle cells, cardiac myocytes, and human endothelial cells (de Crombrugghe et al., 2000; Lundin et al., 2004; Jaulmes et al., 2006). Moreover, the level of mPGES-1 has seemed to be up regulated 10-folds in diabetic patients then the normal healthy individual, suggesting the significant roles of up regulated mPGES-1 expression in development of various pathological conditions (Cipollone et al., 2003b; Sampey et al., 2005; Kosek et al., 2015).

### PGE_2_ (EP) receptor physiological actions and role in inflammation

In past two decades numerous studies have been carried out of knock out mice model to elucidate the physiological functions of EP subtypes in human body. These studies have also been helpful in exploring the specific EP subtypes agonist/antagonist that can be used to innervate, identify and pinpoint the EP sub-types involved in carrying out multifaceted PGE_2_ pathophysiological actions (Ushikubi et al., 1998). For instance in recent study NSAIDs was successfully able to reduce the pyrogenic fever and release of corticotropin-releasing hormone by blocking the EP1 and EP3 signals transduction to hypothalamus (Matsuoka et al., 2003). Moreover, EP receptors play significant role in regulating the ovulation and fertilization process. In has been observed the expansion of cumulus, which is vital for the ovulation and fertilization, is majorly innervated by EP2 (Hizaki et al., 1999). Additionally, Literature suggests that EP1 and EP2 plays significant role is inducing hyperalgesia during inflammation. For instance a recent acetic acid writhing test carried out on rat model has suggested the role of EP1 and EP2 in hyperalgesia induced by rapid heat and pH fluctuations in the body (Hervé et al., 2003). The hypothesis was further cemented by the recent study which stated that pH and heat induced hyperalgesia was significantly reduced by down regulating the expression of capsaicin receptor TRPV1 mainly innervated by release of PGE_2_ and PGI_2_ on EP1 and EP2 receptors (Moriyama et al., 2005). Likewise in the CNS, PGE_2_ mediated EP2 activation escalated the pain sensation and transmission of nociceptive signals in CNS via glycine-induced tonic inhibition of pain neuron in the dorsal horn (Zeilhofer, 2005). In the light of above stated studies it could be inferred that Prostanoids, particularly PGE_2_ plays significant role in mediating inflammation. Moreover, it can also be inferred that pro and anti-inflammatory activity of PGE_2_ are innervated through modulating the EP and IP gene expression on various tissues on the body. For instance recent study suggests that overexpression of EP2 and EP4 has been observed in collagen-induced arthritis rat model, which was also, accompanied by elevated concentration of PGE_2_ at the site of collagen-induced arthritis (Honda et al., 2006). Likewise in another study test samples from the carrageenan- induced paw edema and carrageenan-induced pleurisy revealed overexpression of EP2, EP3, and IP in exudates (Murata et al., 1997). Moreover, there are several studies, which point out toward the role or EP in the development of inflammation and anaphylactic shocks. A recent study suggests that EP3 receptors are fairly distributed on airway epithelium, which upon activation can result in PGE_2_-EP3 pathway activation eliciting strong anaphylactic allergic inflammation (Murata et al., 1997).

## Role of COX-2 and PGE_2_ in various diseases

### Autoimmune diseases

Several pharmacological studies conducted on eicosanoids have given the genetic evidence of PGs and COX-2, in development of autoimmune diseases including rheumatoid arthritis (RA) (Minghetti, 2004; Lucas et al., 2006). In a recent study conducted on mice arthritis model with knocked out cPLA2, COX-2, m-PGES-1 have exhibited significant deceases in inflammatory response in swollen joints. COX-2 mediated intra-articular PGE_2_ production in inflamed joints is carried out by synoviocytes, which is responsible for progression of RA (Akaogi et al., 2006; Shinkai et al., 2008). Moreover, it has been observed that excessive production of PGE_2_ can also produce immunosuppressant effects via suppression of IL-2 production by lymphocytes, by indirectly modulating the activation of CD8^+^ suppressor cells (Demeure et al., 1997).

### Allergic diseases

Allergic reactions are significantly mediated by eicosanoids (Rubin and Mollison, 2007). It has been observed that allergic models with knock out cPLA2, 5-LO, COX-2, and CysLT1 have reduced the frequency and intensity of allergic sign and symptoms (Drazen et al., 1999; Harizi et al., 2008). During the allergic response eicosanoids are produced by monocytes and T-lymphocytes. These eicosanoids are do not impose their effect of immune system directly rather they are responsible for indirectly modulating the system and producing clinical manifestations associated with allergic reaction which includes blood pressure fluctuation, broncho-spasm, diarrhea and fever (Harizi et al., 2008). PGD2, PGE_2_, and PGF2a, IL have no storage space in cells rather they are produced extemporaneously during allergic response. The attachment of allergen with IgE stimulates the PLA_2_ that results in the production of AA. Which is further metabolized by COX/LOX pathway (Peters et al., 1984; Harizi et al., 2008).

### Alzheimer's disease (AD)

Formation of Microglial plague, cytokine induced acute phase reaction and activation of complex cascade are the clinical features of Alzheimer's disease. Significant neuronal damage and worsening of sign and symptoms has been observed with inflammation response (Breitner, 1996; Akiyama et al., 2000; BV and BE, 2000). A recent study on *in vivo* rat model of AD has reported up regulated COX-2 expression and PGE_2_ level present in cerebrospinal fluid. Moreover, the report suggested that increases COX-2 activity in brain has been associated with the AD clinical manifestation including amyloidosis and dementia. Hence it is proposed that early treat with NSAIDs or selective COX-2 can ameliorate or even slow down the clinical manifestation of AD (Weggen et al., 2001; Sciulli et al., 2005).

### Cancer

Several pharmacological studies conducted on eicosanoids have highlighted their role in the development and prognoses of numerous cancers (Wang et al., 2004; Krysan et al., 2006). In a recent study conducted in animal model with knock out cPLA2, COX-1, COX-2, and mPGES-1 have exhibited suppression in tumor development, while rat model will knock out PGD synthase resulted in proliferation of tumor cells (Takaku et al., 2000; Tiano et al., 2002; Kawamori et al., 2005). COX-2 and LOX enzymatic activity and their byproduct have proved to be essential for cancer development of numerous cancers. Biopsy form breast cancer, colon cancer, and prostate have exhibited higher levels of mPGES-1 and COX-2 overexpression. COX-2 mediated PGE_2_ provide safe harbor for the cancer development through promoting angiogenesis, stimulating cellular proliferation, angiogenesis, and removing the cell cycle check points (Öhd et al., 2003; Ding et al., 2005; Paruchuri et al., 2006). Immunosuppression is the most common clinical manifestation associated with tumor development (Sharma et al., 2003). Data have suggested that tumor cell weaken the immune-surveillance via producing excessive amount of immunosuppressive mediator (Avis et al., 2001). Herein the PGE_2_ serve a pseudo-immunosuppressive mediator via obstructing cell differentiation properties of dendritic cell which results is production of uncontrolled undifferentiated cells (Pradono et al., 2002; Edelman et al., 2008).

## Natural COX-2 and PGE_2_ inhibitor past, present and future

The elucidation and isolation of crystal structure COX-2 opened up avenue for new therapeutic options and drug designs (Kiefer et al., 2000; Pouplana et al., 2002). The discovery of COX-2 revolutionized the whole anti-inflammatory treatment, since it was the common perception that unwanted side effects of the NSAIDs are due to inhibition of constitutive role of COX-1. Hence it was proposed that selective COX-2 inhibitors are expected to produce similar therapeutic activity like classical NSAIDs, but with lesser side effects (Ray et al., 2002). However, Rofecoxib, the first selective COX-2 inhibitor was far from being perfect. Clinical trial results suggested that prolong use of rofecoxib can lead to serious cardiovascular complication including cardiomayopathy and ischemic heart failure through disturbing the hemostatic prostacyclin/thromboxane balance (Bing and Lomnicka, 2002). Moreover, a randomized placebo-controlled trial conducted on roficoxib, to study the role of selective COX-2 in prevention of adenomatous polyps raised serious safely issues. The patient treated with selective COX-2 inhibitors exhibited life threatening myocardial infarction symptoms, over the course of 18 months of treatment. This event raise safety concerns for all the members of selective COX-2 inhibitors (Dieppe et al., 2004). However, over the course of two decades several new members of this class including celecoxib, parecoxib, valdecoxib, and Lumiracoxib have come into the market, with claimed gastrointestinal benefits and lacking cardiovascular symptoms (FitzGerald, 2004; Lyon, 2004).

The natural products have served the human kind for thousand of years. For centuries, traditional remedies were on the only source medicine for treating various diseases (Raja et al., 2016). Likewise there are evidences from pre historic times, which suggest the use of traditional remedies for all sort of inflammatory condition. These ethno-pharmacological practices can be dated back to 400 BC, where Greeks used bark of willow tree as a common medical practice to treat inflamed joints and fever. This traditional remedy led to development of Aspirin, the first synthetic plant derived drug to treat rheumatic diseases (Vane, 1971). This discovery further highlighted the importance of natural products in drug discovery and design. In the light of above facts, natural products offer great hope for the discovery of lead compounds with structural diversity and superior efficacy (Polya, 2003). The current review is an effort to highlight the isolates from plant, animal, fungal, and terrestrial and marine algal species with COX-2 and PGE_2_ activity. Since COX-2 derived PGE_2_ production is responsible for progression of numerous inflammatory condition hence it is widely accepted that phytochemical with potent PGE_2_ and COX-2 will exhibit mark analgesic, antipyretic and anti-inflammatory activity.

### Alkaloids

*Berberis* species are used as traditional medicine for treating various inflammatory diseases. Specifically crude roots and bark extracts are used as household remedy for rheumatism, backache and rheumatic fever (Yeşilada and Küpeli, 2002). Numerous studies have suggested the anti-inflammatory activity is due to the abundance of berberine **(1)** (Figure 2), an alkaloid present inside the *Berberis* sp. A recent study conducted on rat model to evaluate the anti-inflammatory activity of *Berberis vulgaris* suggested that berberine **(1)** has exhibited strong anti-inflammatory activity. However, in same study it was reported that treatment with berberine **(1)** is also associated with concentration dependent gastric ulceration. Which led to the conclusion that berbarine share its mechanism of actions with classical NSIADs that produce mark anti-inflammatory activity via inhibiting prostaglandin synthesis that may also be responsible for exhibiting unwanted gastro-intestinal effects (Küpeli et al., 2002). Recent mechanistic study conducted by Kuo et al. (2004) further cemented the COX-2 inhibitory activity of berberine **(1)**. Where pretreated oral cancer cell line OC2 and KB cells with various concentrations (1, 10, and 100 mM) of berberine **(1)** have shown dose dependent PGE_2_ inhibitory activity via suppressing the COX-2 expression. Moreover, in the same study berbarine **(1)** was also able to inhibit activator protein 1 (AP-1), a transcription factor responsible for producing inflammation-mediated cancers. In another study berberine **(1)** exhibited potent apoptotic potential in KB cells via modulating its COX-2 activity. Moreover, berberine **(1)** suppressed Akt phosphorylation and Mcl-1 expression which led to mark COX-2 inhibition (Chi-Li et al., 2005). In light of the above facts it can be concluded that berberine **(1)** can be a therapeutic option in treating inflammation and COX-2 mediated cancer (Fukuda et al., 1999).

**Figure 2:** Structure of alkaloids with potent COX-2 and PGE_2_ inhibitory activity (1) Berberine, (2) Rutaecarpin, (3) evodiamine, (4) Dehydroevodiamine, (5) tryptanthrin, (6) 7′-(3′,4′dihydroxyphenyl)-n-[(4-methoxyphenyl) ethyl] propenamide (Z23), (7) acetylmelodorinol.

Lately a phytochemical analysis was carried out on *Evodia rutaecarpa*, which afforded rutaecarpine **(2)** (Figure 2), an alkaloid with selective COX-2 inhibitory activity. Henceforth, this study was designed to evaluate its effect on PGD_2_ production in bone marrow derived mast cells (BMMC) and its COX-2 mediated PGE_2_ inhibitory activity in HEK293 cells. The results suggested that rutaecarpine **(2)** able to inhibit COX-1 and COX-2 mediated PGD_2_ production in BMMC at a concentration dependent manner with an IC_50_ value of 0.28 and 8.7 μM, respectively. In addition rutaecarpine **(2)** was also able to inhibit COX-2 mediated PGE_2_ production in HEK293 at same concentration range. Moreover, the study conducted by Choi et al. (2006) further cemented the anti-inflammatory activity of *Evodia rutaecarpa's* alkaloids. This study was designed to evaluate the anti-inflammatory activity of rutaecarpine **(2)** and evodiamine **(3)** (Figure 2). Evodiamine **(3)** and rutaecarpine **(2)** significantly inhibited PGE_2_ production in LPS-induced RAW 267.7 cell with an IC_50_ range of 1–10 μM. Moreover, evodiamine was also able to suppress the COX-2 expression via inhibiting NF-κB activation. Likewise, in recent study conducted on *Evodia fructus* have highlighted the anti-inflammatory activity of its major quinazoline alkaloid dehydroevodiamine **(4)** (Figure 2). The results suggested that dehydroevodiamine **(4)** was able to produce mark PGE_2_ and COX-2 inhibition via inhibiting the nuclear factor-kappa B (NF-κB) activity in LPS-induced RAW 264.7 macrophages cells. Therefore, it is strongly suggested that dehydroevodiamine **(4)** can serve as potent anti-inflammatory agent due to its ability to inhibit COX-2 mediated PGE_2_ production in LPS-activated NF-κB (Noh et al., 2006).

*Isatis tinctoria* is widely used by the natives of tropical rain forest as a traditional remedy against all sort of inflammatory conditions (Hamburger, 2002). Recently Danz et al. (2001) evaluated the anti-inflammatory activity of tryptanthrin **(5)** (Figure 2), an alkaloids widely exist in *Isatis* species. The results suggested that tryptanthrin **(5)** was significantly able to inhibit the COX-2 activity with an IC_50_ value (IC_50_ = 64 μM) comparable to that of positive control Nimisulide (IC_50_ = 39 μM). Moreover, similar activity was reported from recent study conducted on novel alkaloid isolated from *Fissistigma cavaleriei* root. The study was designed to evaluate the effect of COX-2 inhibition on angiogenesis of tumor of cells. The results suggested that pretreatment with 8, 16, 32, 64, and 128 μg/ml of compound 1 (name not specified by author) have shown potent dose dependent COX-2 inhibitory activity which led to disruption of newly formed blood vessels in chicken chorio-allantoic membrane. It the light of this study it is suggested that anti-angiogenic property of compound 1 is mainly due to its COX-2 inhibitory activity which can be use as therapeutic option in those tumors where over-expression of COX-2 play significant role (Yang et al., 2012). In another study 7′-(3′,4′-dihydroxyphenyl)-n-[(4-methoxyphenyl) ethyl] propenamide (Z23) **(6)** (Figure 2), an alkaloid isolated from *Fissistigma oldhamii* was evaluated for its anti-inflammatory activity. The results suggested that Z23 has exhibited mark PGE_2_ inhibition via suppressing the COX-2 expression in LPS-induced RAW 264.7 macrophages (Yang et al., 2012). Moreover, Saadawi et al. (2012) reported the similar activity for the acetylmelodorinol **(7)** (Figure 2) isolated from *Mitrella kentia*. The results suggested the acetylmelodorinol was able to inhibit in PGE_2_ in LPS-induced human blood with an IC_50_ value of 19.1 μM. It was proposed that acetylmelodorinol **(7)** exhibited PGE_2_ inhibition via modulating the COX-2 activity. However, more work needs to done on acetylmelodorinol in order to validate this claim.

### Terpenoids

Japanese have used *Acanthopanax kiusianus* Nakai for centuries due to its medicinal activities. *A. kiusianus* is claimed to reduce neurological pain, rheumatism, inflammation of joints, and muscles (Fukuda et al., 2011). However, there were no scientific evidences to these medicinal practices. Until, Suh et al. (2001) conducted a docking study to validate anti-inflammatory activity of *A. kiusianus*. The results suggested that acanthoic acid **(8)** (Figure 3) a novel pimarane diterpene isolated from *A kiusianus* has the potential to inhibit COX-1 and COX-2 at a IC_50_ range of 116.4 and 790.4 μM, respectively. However, more work need to be carried on the plant species in order to validate its claimed anti-inflammatory activity. Likewise, *Acanthopanax trifoliatus* is famous in Southeast Asia, due its wide range of medicinal activity against lung hemorrhages, partial paralysis and neurological pain (Prajapati et al., 2003). Recently, Kiem et al. (2004) conducted phytochemical analysis which afforded one new and three old diterpene glycoside. Out of all the isolated compounds 16aH,17-iso-valerate-ent-kauran-19-oic acid **(9)** (Figure 3), ent-kaur-16-en-19-oic acid **(10)** (Figure 3), and ent-pimara-8(14),15-dien-19-oic acid **(11)** (Figure 3) have shown activity against COX-1 and COX-2 with an IC_50_ value of 0.21, 0.15, and 0.19 μM and for COX-2 with an IC_50_ range of 1.1, 1.2, and 1.5 μM, respectively. The results from this study has provided scientific evidence for the medicinal activity of *A. trifoliatus*, however more animal studies should be carried out in order to validate the claimed medicinal activity (Kiem et al., 2004). Moreover, Kaurenoic acid (ent-kaur-16-en-19-oic acid) **(10)**, diterpenoid isolated from *Aralia continentalis* (*Araliaceae*) root was investigated for its anti-inflammatory activity. Kaurenoic acid was able to significantly reduce the diameter in carrageenan-induced paw edema mice model. Moreover, Kaurenoic acid **(10)** concentration dependently inhibited the PGE_2_ release with an IC_50_ value of 51.73 ± 2.42 μM via suppressing the COX-2 activity in LPS-induced RAW264.7 macrophages with IC_50_ value of 106.09 ± 0.27 μM respectively (Choi R. J. et al., 2011). Likewise in a recent phytochemical analysis carried out on aerial parts of *Artemisia sylvatica* afforded 9 sesquiterpenes. Out of all the isolated compounds arteminolide B **(12)** (Figure 3) was able to suppress NF-κB mediated expression of COX-2 with an IC_50_ value of 7.17 μM. This study was first to report the anti-inflammatory activity of *A. sylvatica* via inhibiting the NF-κB pathway (Jin et al., 2004).

**Figure 3:** Structure of terpiniods with potent COX-2 and PGE_2_ inhibitory activity (8) Acanthoic acid (9)16aH,17-iso- valerate-ent-kauran-19-oic acid, (10) ent-kaur-16-en-19-oic acid, (11) ent-pimara-8(14),15-dien-19-oic acid, (12) Arteminolide B, (13) yaminterriterms B, (14) fomitopinic acid A, (15) Fomitoside, (16) fomitoside F, (17) Manoalide, (18) Scalaradial, (19) Buddledin A, (20) Crocetin monogentibiosyl ester, (21) cyclomargenyl-3-0 -beta-caffeoyl ester, (22) alpha-cyperone, (23) zedoarondiol, (24) curdione, (25) curcumin, (26) eupatolide, (27) koetjapic acid, (28) 3-oxoolean-12-en-30-oic (28), (29) betulinic acid.

*Aspergillus terreus* is a widely distributed thermophilic fungus, can easily be found in soil all around the world. Recently Liaw et al. (2015) has reported to isolate two new polyketide-terpenoid from *A. terreus*. The results suggested that yaminterriterms B **(13)** (Figure 3) significantly inhibited the COX-2 activity with an IC_50_ value of 18.3 μg/ml in LPS-induced RAW 264.7 cells. As mentioned earlier, in past few decades various fungal species have afforded numerous bioactive chemicals with wide range of therapeutic activities. Recent study designed by Yoshikawa et al. (2005) was an effort to explore the natural products with potent anti-inflammatory activity from *Fomitopsis pinicol*. Out of 12 isolated compounds, fomitopinic acid A **(14)**, fomitoside E **(15)**, and fomitoside F **(16)** (Figure 3) were significantly able to inhibit COX-2 activity with an IC_50_ range 0.15–1.15 μM, as compare with positive control indomethacin with an IC50 value of 0.60 μM. Similarly, numerous marine based natural product have gave also interest of the researchers due to their significant anti-inflammatory activity. Specifically, marine sponges are best known for its anti-inflammatory hydroqionones (Glaser and Lock, 1995). In a recent study conducted on *Cacospongia mollior* have afforded two-sesterterpenoid manoalide **(17)** and scalaradial **(18)** (Figure 3). Bio-assay analysis have revealed that both compounds were able to suppress the LPS-induced PGE_2_ production with an IC_50_ value of 10.11 and 21.21 μM in RAW macrophage cells respectively. Hence the results from this study have suggested that marine based products have a huge potential to serve a future lead compound for therapeutic purposes (Potts et al., 1992; Faulkner, 2001). Moreover, in a recent phytochemical analysis carried on Chinese herbal medicine have afforded three new and four known terpinpoids. Out of all the isolated compounds buddle din A **(19)** and crocetin monogentibiosyl ester **(20)** (Figure 3) was able to inhibit COX-2 activity with an IC_50_ value of 13.7, 28.2 and 77.7 μM respectively. Moreover, in the same study buddle din A was also able to demonstrate activity against LOX-5 with an IC_50_ value of 50.4 μM.

*Costus speciosus* is a widely used medicinal plant due to its potent activity against bronchitis, asthma, rheumatisms, inflammation, and fever (Katewa et al., 2004; Saraf, 2010), In recent study Al-Attas et al. (2015) evaluated the anti-inflammatory of its secondary metabolites. It was reported that all the compounds have shown some degree of anti-inflammatory activity. However, 2 new terpinoids were most active against LPS-induced COX-2 mediated PGE_2_ production. Moreover, all tested compounds were also able to reduce the production pro-inflammatory cytokine including IL-1β, IL-6, and TNF-α. Hence this study supports the use of *C. speciosus* as traditional remedy against inflammation associated diseases. Similarly, *Krameria pauciflora* belongs to a small family with merely 17 plant species. However, Mexicans have been using *Krameria pauciflor* for hundreds of years as a traditional medicine against inflammation (Bombardelli et al., 2001; Silva et al., 2001). In recent study of Ramírez-Cisneros et al. (2012) anti-inflammatory activity of *Krameria pauciflor* constituents were determined. Out of all the isolated compounds cyclomargenyl-3-O-β-caffeoyl ester **(21)** (Figure 3) reported the most significant (*p* < 0.05) activity against COX-2 and PLA_2_ with an IC_50_ value of 10 μM.

Likewise *Cyperus rotundus* is an Asian medicinal plant used in Chinese traditional medicine for treating various inflammatory conditions. In recent work of Jung et al. (2013) the anti-inflammatory activity of α-cyperone **(22)** was evaluated on LPS induced RAW macrophage cells (Figure 3). α-cyperone **(22)** significantly inhibited the PGE_2_ production via inhibiting the COX-2 activity in LPS induced RAW macrophage cells. Moreover, pretreatment with α-cyperone also suppressed the NF-κB activation and nuclear translocation in LPS induce cells. Hence suggesting that anti-inflammatory activity α-cyperone is related with its ability to suppress the transcriptional activity of NF-κB. Likewise, a sesquiterpene lactone zedoarondiol **(23)** (Figure 3) isolated from *Curcuma heyneana* rhizome shared similar anti-inflammatory activity. Zedoarondiol **(23)** exhibited dose dependent inhibition of IL-1β, IL-6, and TNF-α in LPS-induced macrophage cells. Moreover, expression of COX-2 and iNOS was also down regulated with the pretreatment of Zedoarondiol **(23)**. Further mechanistic study revealed that Zedoarondiol **(23)** blocked the activation and transmigration of NF-κB to the nucleus and decreasing the phosphorylation of IκB kinase, which probably let to suppression of COX-2 expression (Cho et al., 2009). Similarly, in an effort to find natural products with anti-inflammatory activity, curdione **(24)** (Figure 3) sesquiterpenoids isolated form *Curcuma zedoaria* was evaluated against LPS-induced PGE_2_ production in RAW macrophage cells. Curdione **(24)** dose dependently inhibited the PGE_2_ production with an IC_50_ value of 1.1 μM. Further mechanistic study revealed that curdione **(24)** was able to decrease the PGE_2_ production via suppressing the COX-2 mRNA expression (Cho et al., 2009). In another study, *Curcuma longa* from Zingiberaceae family exhibited similar anti-inflammatory activity. It was observed that pre-treatment with 80 μg/ml of curcumin **(25)** (Figure 3) suppressed cell proliferation associated gene products (COX-2, cyclin D1, and c-myc) which led to the suppression of anti-appoptotic proteins including IAP1, IAP2, X-chromosome-linked IAP, Bcl-2, Bfl-1/A1 via blocking the TNF-α induced NF-κB activation. In a recent study conducted on *Inula britannica* to evaluate its anti-inflammatory reported similar NF-κB activity. The results have shown that eupatolide **(26**) (Figure 3) sesquiterpene lactone have potentially inhibited NO and PGE_2_ release and COX-2 and iNOS mRNA expression in a concentration dependent manner. Moreover, it was concluded that suppression of gene expression was due its ability to block NF-κB activation, IkB degradation, MAPKs pathway and suppress Akt in LPS-stimulated RAW264.7 cells (Lee et al., 2010).

Annonaceae is among the largest planet family with more than 3,000 species. Many of its species are famous in regions of rain forest due to wide range of medicinal activities (Attiq et al., 2017). *Dillenia serrate* is also popular among Malaysian peninsular region due to its medicinal activity against internal hemorrhage, rheumatism, generalized body pain and inflammation (Jain, 1994; Panda, 2004). However, there are very few study conducted on this species to support its medicinal use. Hence forth in a recent study Jalil et al. (2015) evaluated a three triterpinoid koetjapic acid **(27)**, 3-oxoolean-12-en-30-oic **(28)**, and betulinic acid **(29)** (Figure 3) isolated from the *D. serrate*. All the compounds exhibited significant concentration-dependent inhibitory effects on PGE_2_ production with IC_50_ values of 1.05, 1.54, and 2.59 μM respectively, as compared with the positive control, indomethacin (IC_50_ = 0.45 μM). Moreover, it was proposed that compounds were able to inhibit the PGE_2_ release via modulating the COX-2 activity. However, more work need to be carried out on *D. serrate* in order to support the proposed COX-2 inhibitory mechanism. Likewise, *Euphorbia nivulia* belong to the Euphorbia family, which is considered as the largest family of this genera with more than 1,000 plant species. Due to its medicinal properties it has been used in Ayurveda medicine for treating rheumatism and bronchitis (Rates, 2001; Ernst et al., 2015). In late study conducted to determine the PGE_2_ inhibitory activity of *E. nivulia* isolates suggested that 7-angeloyl-12-acetyl-8-methoxyindol **(30)** (Figure 3) have shown significant PGE_2_ inhibition with an IC_50_ of 0.003 μM, which is comparable to the positive control Celecoxib (IC_50_ = 0.05 μM) (Ravikanth et al., 2002).

### Stilbenes

Several plant species have been reported to have stilbenoids, a unique class of phytochemical with wide range of bioactivity (Surh, 1999). In last two decades several reports have highlighted the anticancer activity of well-established chemo-preventive secondary metabolite resveratrol **(31)** (Figure 4) (Jang et al., 1997; Bhat and Pezzuto, 2002). In current study usefulness of resveratrol (31) was evaluated in neurodegenerative diseases via utilizing its ability to suppress the inflammation via blocking the cyclooxygenase pathway and its components (COX and PGs). Results suggested that pretreatment with 1–50 μM resveratrol (31) in LPS induced primary microglial cell significantly (*p* < 0.05) down regulated the expression of COX-1, COX-2, and mPGES-1 in a concentration dependent manner. Hence suggesting the usefulness of resveratrol (31) in treating neurodegenerative diseases where overactive cyclooxygenase pathway plays significant role in disease progression (Candelario-Jalil et al., 2007). Moreover, finding from the current study has further cemented the efficacy of resveratrol (31) in neurodegenerative diseases, (Li et al., 2012) which suggest that resveratrol (31) was able to inhibit the expression of COX-2 and mPGES-1 in LSP induced microglial cell in a concentration dependent manner. In the same study it was also observed resveratrol facilitates the non-amyloidogenic cleavage of the amyloid precursor protein which plays significant role in the clearance of amyloid beta-peptides involved in neuronal damage.

**Figure 4:** Structure of stilbenes with potent COX-2 and PGE_2_ inhibitory activity (31) transresveratrol, (32) aiphanol, (33) isorhapontigenin, (34) oxyresveratrol, (35) artocarpesin, (36) pinosylvin, (37) desoxyrhapontigenin.

In a recent study phytochemicals of *Aiphanes aculeata* were evaluated for ability to suppress the COX-2 expression in various cancer cells line. It was reported that among all the isolated compounds aiphanol **(32)** and isorhapontigenin **(33)** (Figure 4) significantly inhibited COX-1 (IC_50_ = 1.9 and 1.5 μM) and COX-2 (IC_50_ 9.9 and 6.2 μM) in a concentration dependent manner. The results suggested that aiphanol **(32)** and isorhapontigenin **(33)** (Figure 4) could be possible alternative therapeutic option for cancers ailment, as COX-2 over expression plays significant role in cancer development and progression (Lee et al., 2001). In another *in vitro* study oxyresveratrol **(34)** and artocarpesin **(35)** (Figure 4) isolated from *Artocarpus heterophyllus*, showed promising anti-inflammatory activity. Oxyresveratrol **(34)** and artocarpesin **(35)** inhibited the NO and PGE_2_ production in LPS-induced RAW 264.7 cells via suppressing the expression of the iNOS and COX-2 respectively. Which signify their role as a potential therapeutic candidate for treating inflammation mediated diseases (Fang et al., 2008).

In Chinese traditional medicine root and leaves of *Hovenia dulcis* are used as a traditional remedy to treat peptic ulcers, liver toxicity and inflammation (An et al., 1999; Kim et al., 2014). However, there were lack of scientific evidence for these traditional practices until Lim et al. (2015) carried out anti-inflammatory studies on the secondary metabolites of *H. dulcis* to validate this claim. The results suggested that methanol extract of *H. dulcis* reduced the release and production of PGE_2_, IL-4, and TNF-α in a concentration dependent manner. Moreover, in the same experiment the methanolic extract of *H. dulcis* suppressed the COX-2 expression via blocking the NF-κB activation. The phytochemical analysis of *H. dulcis* extract revealed that pinosylvin **(36)** (Figure 4) was mainly responsible for the producing the inhibitory activities of methanolic extract. Similarly *Rheum undulatum*, another plant species from Chinese traditional medicine was subjected to the phytochemical analysis, which afforded desoxyrhapontigenin **(37)** (Figure 4). Bioassay analysis showed that desoxyrhapontigenin **(37)** significantly decreased the NO and PGE_2_ production at a concentration range of 10–50 μM. Additionally, it was observed that desoxyrhapontigenin was also able to suppress the expression of iNOS and COX-2 by blocking the LPS- induced NF-κB activation in RAW macrophage cells (Choi et al., 2014). This study suggests that desoxyrhapontigenin **(37)** has the potential to resolve inflammation by suppressing the expression of inflammatory mediators via blocking the transcriptional activity of NF-κB.

### Flavonoids

*Artemisia feddei* is widely used in African countries due to its ornamental and medicinal uses (Kim et al., 1999). The bark and leave decoction has been used as traditional remedy for digestive and inflammatory disorder (Kang et al., 1999). In recent study, Kim et al. (2004) reported the anti-inflammatory activity of scopoletin **(38)** (Figure 5) isolated from *A. feddei*. Pretreatment with 1–50 μg/ml of scopoletin (38) was able to significantly inhibit the production of PGE_2_, TNF-α, IL-1β, and IL-6 in a concentration dependent manner. Further studies suggested that scopoletin (38) inhibited the PGE_2_ production via inhibiting the LPS-induced COX-2 activity in RAW 264.7 macrophages. Likewise, Noreen et al. (1998) evaluated the anti-inflammatory activity of the flavonoids obtained from various medicinal plants including *Atuna racemosa, Syzygium corynocarpum, Syzygium malaccense*, and *Vantanea peruviana*. Among all the isolated flavonoids (+)-catechin **(39)**, (+)-gallocatechin **(40)**, 4′-*O*-Me-*ent*-gallocatechin **(41)**, ouratea-catechin **(42)**, and proanthocynidin A **(43)** (Figure 5) demonstrated inhibition of COX-2 activity with an IC_50_ range from 3.3 to 138 μM. These results suggested that medicinal activities of these plants extracts were due to the COX-2 inhibitory activity of its flavonoids. Unlike the previous studies conducted on perennial plant species, Ogundaini et al. (1996) focused on a parasitic plant *Sarcophyte piriei*, which proliferates on the roots of Acacia species. There are several reports which signifies the medicinal activity of this parasitic species against abdominal pain, toothache, and burses (Pongprayoon et al., 1991; Farah and Samuelsson, 1992). However, the phytochemical and pharmacological profile of this plane specie is not well-established. Hence Ogundaini et al. (1996) designed study to evaluated the phytochemistry and anti-inflammatory activity of *S. piriei*. The phytochemical analysis revealed two new flavonoid c **(44)** and diinsinin **(45)** (Figure 5) and pharmacological screening suggested that both compounds had excellent PGE_2_ inhibitory activity with IC_50_ values 9.20 and 13.14 μM, respectively. Moreover, upon further analysis both flavonoids suppressed PAF induced exocytosis with IC_50_ values 49 and 39 μM. In conclusion it was proposed that these compounds were able to inhibit PGE_2_ production via attenuating the COX-2 activity in LPS induced RAW macrophage cells. Likewise, in a recent study anti-inflammatory activity of *Chrysopogon aciculatis* was also evaluated in LPS-induced RAW macrophage 264.7 cells. The phytochemical analysis of acetone fraction of *C. aciculatis* afforded aciculatin **(46)** (Figure 5). The bioassay results demonstrated potent PGE_2_ and NO inhibitory activity of aciculatin **(46)** with an IC_50_ range of 1–10 μM. Aciculatin **(46)** was also able to suppress the expression of iNOS and COX-2 via inhibiting the activation and translocation of NF-κB in LPS-induced RAW 264.7 cells. Moreover, aciculatin **(46)** was also able to suppress IκB kinase activation and phosphorylation of MAPKs. Hence suggested the anti-inflammatory activity of aciculatin **(46)** was due to its ability to suppress the transcriptional activity of NF-κB and MAPKs (Hsieh et al., 2011). Francis et al. (2004) reported the similar COX-2 suppressing activity of Kaempferol, isolated from Easter lily (*Lilium longiflorum*) flowers. In lipid peroxidation inhibitory assay kaempferol **(47)** strongly inhibited the COX-2 activity by 36.9% at 80 ppm. While it was observed that the inhibitory activity was not concentration dependent since in the same experiment kaempferol **(47)** inhibited COX-2 activity by 37% at 1 ppm, while 100% COX-2 inhibition was observed at 10 ppm respectively. However, in another study delphinidin 3-O-beta-galactopyranoside, cyanidin 3-O-beta-galactopyranoside, and pelargonidin 3-O-beta-galactopyranoside, three novel anthocyanins failed to show any significant anti-inflammatory activity. It was reported that all the tested compounds were only able to inhibit COX 1 by 9.23, 11.71, and 7.66% with an IC_50_ values ranging 40–170 μM. While isolated compounds merely inhibited COX-2 activity by 7.65, 12.46, and 7.38% at the same concentrations. Hence anti-inflammatory activity of these compounds were considered insignificant, as compare to the positive control used in the experiment (Naproxen) (Seeram et al., 2002). Moreover, in a recent study carried out on in order to investigate the mechanism to action through which bacterial endotoxins and cytokines induce the gene expression of COX-2 and mPGES-1, which are directly related to the increases turn over of PGE_2_ in macrophages and other tissues. Out of 24 naturally occurring flavonoids tested kaempferol **(47)** most significantly suppressed the LPS induced COX-2 and mPGES-1 with an IC_50_ value of 1.89 and 5.81 μM, as compare to Celecoxib (IC_50_ 1.11 and 4.98) known selective COX-2 inhibitor (Hämäläinen et al., 2011). In order to explore the natural product with anti-inflammatory activity, gigantol **(48)** (Figure 5) isolated from *Cymbidium goeringii* was evaluated against PGE_2_ and NO production in LPS induced RAW 264.7 cells. The results indicated that gigantol **(48)** inhibited NO and PGE_2_ production in a concentration dependent manner. In addition gigantol **(48)** reduced the production and expression of major pro-inflammatory cytokines including TNF-α, IL-1 α, and IL-6. Moreover, gigantol **(48)** also suppressed COX-2 and iNOS expression via blocking the LPS-induce NF-κB activation in a concentration dependent manner. Hence it was proposed that gigantol **(48)** was able to suppress the gene expression of COX-2 and iNOS via blocking the transcriptional activity of the activation of NF-κB. Likewise, Hiermann et al. (1998) evaluated the anti-inflammatory activity of myricetinglucuronide **(49)** (Figure 5) on acute (carrageenan) and chronic (adjuvant arthritis) rat model. COX-2 inhibitory activity was evaluated on perfused rabbit ear. myricetinglucuronide **(49)** was able to reduce inflammation in both acute and chronic inflammation model with an ED_50_ value of 15 and 150 μg/kg, respectively. Pretreatment with 1 μg/ml myricetinglucuronide **(49)** significantly reduced the production of PGI_2_, PGE_2_, and PGD_2_ in perfused rabbit ear. Moreover, myricetinglucuronide **(49)** was also able to suppress the activity of COX-1 and COX-2 with IC_50_ values 9.2 and 2.4 μM, respectively. This study highlighted the anti-inflammatory of myricetinglucuronide in both *in-vivo* and *in-vitro* models signifying the myricetinglucuronide **(49)** as potential therapeutic option for resolving inflammation.

**Figure 5:** Structure of flavanoids with potent COX-2 and PGE_2_ inhibitory activity (38) scopoletin, (39) (+)-catechin, (40) (+) gallocatechin, (41) 4′−0-Me-ent- gallocatechin, (42) ouratea-catechin, (43) proanthocynidin A, (44) flavonoid c, (45) diinsinin, (46) aciculatin, (47) kaempferol, (48) gigantol, (49) myricetinglucuronide, (50) genistein, (51) anthocyanin, (52) tectorigenin, (53) tectoridin, (54) morusin, (55) kuwanon C, (56) sanggenon B, (57) sanggenon C, (58) sanggenon D, (59) wogonin, (60) oroxylin A, (61) baicalein.

Soya bean has been reported to have anti-cancer activity due to presence of genistein **(50)** (Figure 5). Ye et al. (2004) tested genistein **(50)** on a human oral squamous carcinoma line (SCC-25) for the evaluation of anti-cancer potential in COX-2 mediated cancers. The results demonstrated that genistein **(50)** have shown significant cytotoxic activity in both cancer cell line, however it failed to exhibit apoptotic potential in the same study. Moreover, genistein **(50)** also inhibited the enzymatic activity and expression of COX-2 in a dose dependent manner. This study suggests that genistein can serve as potential chemo-protective agents in COX-2 mediated cancers. In another phytochemical study conducted on soya bean afforded anthocyanin **(51)** (Figure 5), a flavanoid with potent anticancer activity (Wang and Stoner, 2008). It was observed that pretreatment with anthocyanin **(51)** exhibited significant reduction in PGE_2_ production in LPS-induced human keratinocyte. Moreover, anthocyanin also blocked the activation of NF-κB and PI3 kinases in UVB exposure human keratinocyte cells. Likewise, Pan et al. (2008) reported the similar activity for two flavonoids, tectorigenin **(52)** and tectoridin **(53)** (Figure 5) isolated from *Iris domestica*. The current study was designed to evaluate the anti-inflammatory activity of these two flavonoids in LPS induced/interferon-γ induced RAW 264.7 macrophage cells. Tectorigenin **(52)** significantly inhibited the production of NO and PGE_2_ through suppressing the expression of iNOS and COX-2 in a concentration dependent manner. Moreover, the pretreatment with tectorigenin **(52)** was also able to block the activation of NF-κB with an IC_50_ value comparable to that of positive control genistein.

Prenylated flavonoids are widely distributed flavonoids with a combination of 1,1-dimethylallyl, an isoprenyl unit a geranyl unit attached together in one structure., Chi et al. (2001b) managed to isolate 19 prenylated flavonoids from *Morus alba* and then evaluated their inhibitory activity against COX-1, COX-2, and 5-LOX. The results suggested that among all the tested flavonoids morusin (54), kuwanon C (55), sanggenon B (56), and sanggenon C (57) (Figure 5) had shown significant inhibitory activity against COX-2 with an IC_50_ value ranging 73–100 μM. However, most of the compounds were more active (IC_50_ = 0.1 to 1 μM) against COX-1 rather then COX-2, hence making them inappropriate for therapeutic use due to gastrointestinal effects associated with COX-1 inhibition. Another study suggested that sanggenon D (58) and B **(56)** (Figure 5) isolated from *Morus mongolica* exhibited similar COX-1 and COX-2 activity with IC_50_ values of 59 and 42 μM for COX-1 and 73 and 100 μM for COX-2 inhibition. Likewise, screening of bioactive isolates carried out by Huang et al. (2016) to establish novel method of orthogonal projection to latent structure and modified principal component analysis revealed that wogonin **(59)** and oroxylin A **(60)** (Figure 5), major component of *Scutellaria baicalensis* significantly inhibited the PGE_2_ production in RAW 264.7 macrophages. Furthermore, similar activity was reported by another study carried out by Fernando et al. (2016) to evaluate the anti-inflammatory activity of baicalein **(61)** (Figure 5) from marine source. The results from this study suggested that baicalein **(61)** exhibited anti-inflammatory activity via modulating the gene expression of major inflammatory mediators including IL-1, MCP1, COX-2. In the same study baicalein **(61)** was also able to suppress the activity of anti-apoptotic proteins including cIAP-1, cIAP-2, and FLIP. Moreover, it was suggested that the reported activity was due to the inhibition of TNF-a induced NF-κB, p65 nuclear translocation and inhibition of phosphorylation and degradation of IkBa.

### Saponins

*Artemisia capillaris* is widely used plant species all around the world to treat pain, inflammation and alcohol induced liver toxicity (Bora and Sharma, 2011; Joshi, 2013). A recent study was carried out to evaluate the anti-inflammatory and analgesic activity of capillarisin **(62)** (Figure 6), a major lignin isolated from *A. capillaris*. The major scope of this study was to evaluate the capillarisin **(62)** activity against MyD88/TIRAP, iNOS, and COX-2 at therapeutic concentrations. It was observed that pretreatment with capillarisin **(62)** significantly inhibited the LPS- induced activation of NF-κB, Akt, and MAPKs mediated inflammatory genes. Moreover, it was also observed that pretreatment with capillarisin was able to reduce the expression of COX-2 and iNOS in LPS-induced RAW 264.7 macrophage cells. In the same study, capillarisin **(62)** also significantly blocked the activation of p-JNK, p-p38, p-ERK, and p-Akt. Hence it was concluded form the present study that the potent anti-inflammatory activity of capillarisin **(62)** was via inhibiting the activation pathways responsible for promoting the activity of inflammatory mediators (Khan et al., 2013). Moreover, a similar study was carried out on an ornamental plant species *Kalopanax pictus*, to evaluate the anti-inflammatory activity of its constituents. Out of all the tested compounds it was observed that monodesmosides **(63)** (Figure 6) and kalopanxsaponin-A **(64)** (Figure 6) most significantly inhibited the NO, PGE_2_, and TNF-α production in LPS- induced RAW 264.7 macrophage cells (Kim Y. K. et al., 2002).

**Figure 6:** Structure of saponins with potent COX-2 and PGE_2_ inhibitory activity (62) capillarisin, (63) monodesmosides, (64) kalopanxsaponin-A, (65) ginsenosides, (66) saponin prosapogenin D methyl-ester, (67)buddlejasaponin I.

Araliaceae family consists of numerous species with potent medicinal activities. Ginseng is most widely consumed medicinal plant from this plant family due to its medicinal activities (Corbit et al., 2005; Park et al., 2005). Ginseng can be used as fresh, dried (white ginseng) or peeled form (red ginseng). However, recent studies have suggested that all forms of ginseng have equal medical activity irrespective of their mode of administration or part used (Kang et al., 2005; Volate et al., 2005). There are several reports which suggest the anti-inflammatory activity of ginseng, including most recent study of Ichikawa et al. (2009) reported that ginsing extract and ginsenosides **(65)** (Figure 6) were able to inhibit the activation of NF-κB and MAPKs. Moreover, ginsenosides **(65)** exhibited potent activity against PGE_2_ and NO via suppressing the COX-2 and iNOS activity in LPS induced macrophage cells. Moreover, in another study conducted to evaluate the anti-inflammatory activity of ginsenosides **(65)** suggested that pretreatment with ginsenosides **(65)** led to down regulation of COX-2 in a concentration dependent manner. Further mechanistic study revealed that ginsenosides **(65)** was able to pull out this activity via suppressing the transcriptional property of NF-κB (Hofseth and Wargovich, 2007). Likewise in another report ginsenoside **(65)** was evaluated for its anti-inflammatory in neurodegenerative disorder including Parkinson diseases. The results suggested that ginsenoside **(65)** was able to reduce the PGE_2_ and NO production via suppressing the COX-2 and iNOS expression hence signifying its importance in treating those neurodegenerative diseases where excessive activity of PGE_2_, NO, and COX-2 plays significant role (Zhang et al., 2006).

*Platycodon grandiflorum* belong to Campanulaceae family and the root this species (*Platycodi Radix)* is widely consumed all around the world as a traditional medicine for lungs infection and ocular inflammation (Ahn et al., 2005; Srivastava et al., 2005). These traditional practices are consistent with the existence of high content of saponin present inside this species (Shin et al., 2002). In a recent study new saponin prosapogenin D methyl-ester **(66)** (Figure 6) isolated form *Platycodi radix* and was evaluated for possible anti-inflammatory activity. It was observed that prosapogenin D methyl-ester **(66)** was able to reduced the biosynthesis of NO and PGE_2_ in a concentration dependent manner. Furthermore, D methyl-ester significantly down regulated COX-2 and iNOS expression via completely blocking the activation of NF-κB in LPS induced RAW macrophage 264.7 cells (Chung et al., 2008). Similar activity was reported for new saponins buddlejasaponin IV **(67)** (Figure 6) isolated from *Pleurospermum kamtschaticum*. Where buddlejasaponin IV **(67)** potentially inhibited the production of PGE_2_, TNF-α, and NO in LPS induced RAW 264.7 macrophage cells.

### Fatty acids

*Daucus carota* is most widely consumed vegetable around the world. Some parts of the world use it as ornamental medicine for digestive disorders, cardiovascular disorders, epilepsy, and infertility (Momin et al., 2003). Recent studies have suggested that high content of essential oils present inside the carrot are responsible for the most of the medicinal activities. Momin et al. (2003) designed a study to determine the anti-inflammatory activity of essential oils isolated from *D.carota*. The results suggested that 2,4,5-trimethoxybenzaldehyde **(68)**, oleic acid **(69)**, and trans-asarone **(70)** (Figure 7) had inhibited the COX-2 activity by 52.69, 68.41, and 64.39%. While all three compounds did not show any significant activity against COX-1. In conclusion, 2,4,5-trimethoxybenzaldehyde **(68)** most significantly inhibited COX-2 in a concentration dependent manner with an IC_50_ value of 100 μg/ml. Likewise form prehistoric times humans have been using mushrooms in daily routine due to their nutritional and medicinal value. One of the most widely consumed mushrooms includes *Grifola frondosa*, which is commonly referred as hen of the woods due to characteristic shape and texture. *G. frondosa* is also one of the main ingredients in Chinese traditional medicine prepared for treating hemorrhoids (Huang and Xie, 1988), gonorrhea (Mizuno and Zhuang, 1995), diabetes (Kubo et al., 1994), neuralgia, and arthritis (Mizuno and Zhuang, 1995). A study by Zhang et al. (2002) was designed to evaluate the potential anti-inflammatory activity of essential oils isolated from *G. frondosa*. It was observed that hexane fraction consisting ergosterol **(71)**, ergostra-4,6,8(14),22-tetraen-3-one **(72)**, and 1-oleoyl-2-linoleoyl-3-palmitoylglycerol **(73)** (Figure 7) has significantly inhibited the COX-1 activity by 98, 37, and 67% at 250 μg/ml. Likewise upon further analysis it was revealed that all the compounds were also able to inhibit COX-2 activity by 99, 37, and 70% at 250 μg/ml, respectively. This study provides evidence of bioactive compounds responsible for producing medicinal activities against inflammatory conditions. Moreover, a recent at study by Wang et al. (2017) further highlighted the anti-inflammatory activity of edible mushroom, which led to the isolation of eburicoic acid **(74)** (Figure 7) from *Laetiporus sulphureus*. The study demonstrated that eburicoic acid **(74)** was able to reduce the PGE_2_ and NO production via suppressing the expression of iNOS and COX-2 in LPS-induced RAW 264.7 macrophage cells. Moreover, it was observed that eburicoic acid (74) significantly inhibited the production of TNF-α, IL-6, and IL-1β and down regulated the expression of PI3k, Akt, mTOR, and NF-κBp65. Hence suggesting that eburicoic acid **(74)** has potent anti-inflammatory activity via suppressing the inflammatory pathways and inhibiting the production of pro-inflammatory cytokines (Wang et al., 2017). Moreover, Paul et al. (2006) reported the similar activity for the 13-(S)-hydroxy-9Z,11E-octadecadienoic acid [(S)-coriolic acid **(75)** (Figure 7) isolated from *Hernandia ovigera* L. The results suggested that 13-(S)-hydroxy-9Z,11E-octadecadienoic acid [(S)-coriolic acid (75) shown selective COX-2 inhibition with an IC_50_ Value of 0.30 μM. However, it was observed that upon increasing the concentration 13-(S)-hydroxy-9Z,11E-octadecadienoic acid [(S)-corioli acid (75) have lost its COX-2 selectivity and also exhibited COX-1 inhibition at concentrations > 100 μM. Moreover, it has the tenacity to suppress the expression of iNOS, COX-2, IL-6, and TNF-a by blocking the activation of NF- and AP-1 activator protein. Furthermore, phytochemical analysis of *Hernandia ovigera* afforded palmitic acid **(76)**, oleic acid **(77)**, linoleic acid **(78)**, linolenic acids **(79)** (Figure 7). This study was designed to evaluate the anti-inflammatory of fatty acid that make up the major composition of *Hernandia ovigera*. All the compounds have shown significantly inhibited the COX-2 activity in a concentration dependent manner with an IC_50_ range of l0.5 to 23.0 μM (Bauer et al., 1996).

**Figure 7:** Structure offatty acids with potent COX-2 and PGE_2_ inhibitory activity (68) 2,4,5-trimethoxybenzaldehyde, (69) oleic acid, (70) trans-asarone, (71) ergosterol, (72) ergostra-4,6,8(14),22-tetraen-3-one, (73) 1-oleoyl-2-linoleoyl-3-palmitoylglycerol, (74) eburicoic acid, (75) 13-(S)-hydroxy-9Z,11E-octadecadienoic acid [(S)-coriolic acid, (76) palmitic acid, (77) oleic acid, (78) linoleic acid, (79) linolenic acids.

### Miscellaneous compounds

*Acanthopanax species* have been used in far East-Asian countries to cure rheumatoid arthritis and diabetes mellitus (Kim and Hahn, 1981; Lee S.-H. et al., 2003). A recent study was carried out to evaluate the anti-inflammatory activity of the lignins isolated from *Acanthopanax chiisanensis*. It was observed that out of five lignins isolated, taiwanin C **(80)** (Figure 8) dose dependently inhibited the PGE_2_ production with an IC_50_ value of 0.12 μM while other four lignin failed to show any activity at given concentrations (Lee et al., 2005). Likewise balanophonin **(81)** (Figure 8), a neolignin isolated from *Firmiana simplex* was evaluated for its ability to reduce neuro-inflammation. This study suggested that balanophonin **(81)** reduced the production of TLR4, NO, PGE_2_, IL-1β, and TNF-α in LPS induced BV2 cells. Moreover, it was also observed that pretreatment with balanophonin also dose dependently suppressed iNOS, COX-2, and MAPKs expression. In the light of this study it could be inferred that balanophonin has the potential to reduce the neuronal cell death by inhibiting microglial activation (Lim et al., 2017). Likewise, *Withania somnifera* is an ever green shrub extensively used in Ayurvedic medicine for treating adenopathy, arthritis, inflammations, and rheumatism (Thakur et al., 1989; Rasool and Varalakshmi, 2006). Withanolides are a specific class of compounds associated with *W. somnifera*, which is responsible for carrying out above stated medicinal activities (Ray and Gupta, 1994). In a recent study withanolide glycosides and withanolided isolated from *W. somnifera* were subjected to anti-inflammatory evaluation. Out of all the isolated compounds sitoindoside IX **(82)** (Figure 8) most significantly inhibited the COX-2 activity with an IC_50_ value of 100 mg/ml. while rest of the compounds exhibited non-selective COX inhibition. Likewise, in anti-proliferative study conducted by Mulabagal et al. (2009) reported similar activity for the withanolide sulfoxide **(83)** (Figure 8) isolated from *W. somnifera*. It was observed that withanolide sulfoxide selectively inhibited COX-2 activity by 60% with an IC_50_ value of 100 μM. Moreover, upon further evaluation withanolide sulfoxide **(83)** have also shown potent anti-proliferative activity in various cancer cell lines [human gastric (AGS), breast (MCF-7), central nervous system (SF-268), and colon (HCT-116)] with an IC_50_ range of 0.74–3.63 μM. It was concluded form the study that COX-2 mediated anti-proliferation was responsible for the cytotoxic activity of withanolide sulfoxide (83) (Mulabagal et al., 2009). Moreover, gingerol **(84)** (Figure 8) is polyphenolic compound, which can be found in majority of Zingiberaceae species. A study was designed to evaluate the effect of gingerol on streptozotocin induced Alzheimer diseases *in vivo* by using whiskers rat model. The basic purpose of the study was to determine that whether the treatment with gingerol can to reduce the inflammation and improve the cognitive impairment in sporadic Alzheimer's disease in whiskers rat model. The results suggested that pretreatment with 10 and 20 mg/kg bwt significantly reduce the α-, β- secretases, APH1a and COX-2 levels, which resulted in the improvement of cognitive behaviors (El Halawany et al., 2017). Likewise similar activity was reported for two styryllactone, altholactone **(85)** and (+)-goniothalmin **(86)** (Figure 8) isolated from *Alphonsea javanica*. It was concluded form the current study that both compounds significantly reduced the LPS-induced NO production, phosphorylation of IKB alpha, and also down regulated the gene expression of iNOS and COX-2 (Johnson et al., 2013). Moreover, diglyceride **(87)** from *Amaranthus tricolor* were also able to inhibit the COX-1 enzyme by 78, 63, and 93%, respectively and the COX-2 enzyme by 87, 74, and 95%, respectively (Jayaprakasam et al., 2004). However, due to their non-selective COX activity, it is expected that use of these diglyceride **(87)** might be associated with undesirable gastrointestinal effects, which limits its use as therapeutic application. Ligustilide **(88)** (Figure 8), phthalide derivative from *Angelica tenuissi* was also subjected to anti-inflammatory evaluation. The bioassay results demonstrated that Ligustilide (87) has potent anti-inflammatory activity by modulating NF-κB and MAPK pathways, which led to the suppression of LPS-induced iNOS and COX-2 expression at both mRNA and protein levels. Furthermore, Ligustilide **(88)** additionally inhibited the phosphorylation of IkBa and p38 mitogen-activated protein kinase in a dose dependent manner (Chung et al., 2012). Bruceine D **(89)** (Figure 8), belong to unique class of compound, which is mostly predominant in Simaroubaceae family. Till this date the pharmacological profile on this class is yet to be established. However, in recent study bruceine D showed significant inhibitory activity against COX-2 with an IC_50_ value of 20.6 μM demonstrating the anti-inflammatory potential of this unique class (Su et al., 2002). Likewise corresponding activity was observed in a study conducted on handelin **(90)** (Figure 8), duaianolide dimer isolated from *Chrysanthemum boreale*. It was observed that handelin **(90)** suppressed NO and PGE_2_ activity via suppressing the iNOS and COX-2 expression in LPS-induced RAW 264.7 macrophage cells. In addition, pretreatment with handelin **(90)** also deceased the production of IL-1β and TNF-α in a dose dependently manner. Further mechanist study revealed that handelin **(90)** also inhibited the activation and translocation of NF-κB into the nucleus, which is in complete conjunction with the suppression of COX-2 and iNOS activity.

**Figure 8:** Sturcture of miscellaneous with potent COX-2 and PGE_2_ inhibitory activity (80) taiwanin C (81), balanophonin (82), sitoindoside IX (83), withanolide sulfoxide (84), gingcrol, (85) altholactone (86), goniothalmin (87), diglyccride (88), ligustilide (89), bruceine D (90), bandelin (91), guggulstcrone (92), isoliquiritin (93), isoliquiritigenin (94), sphondin (95), 4-Methoxyhonokol (96), Schisandrin (97), bocravinone B.

*Commiphora mukul* resins have gain great importance in Ayurvedic medicine due to its wide range of medicinal properties (Craig, 1997). It has been use by Indians for centuries for treating arthritic pain, inflammation, high cholesterol, and osteoarthritis (Gujral et al., 1960; Sharma, 1977; Sinal and Gonzalez, 2002; Urizar and Moore, 2003). Recent studies have shown that guggulsterone **(91)** (Figure 8) isolated from *Commiphora muku* were able to block the activation of NF-κB in TNF-α induced epithelial and leukemia cells. In addition guggulsterone **(91)** also suppressed the phosphorylation and consequent degradation of IκBα, which eventually led to the suppression of inflammatory genes responsible for the activity of MMP-9, COX-2, and VEGF (Shishodia and Aggarwal, 2004). In another study pretreatment with guggulsterone **(91)** blocked the NF-κB activation, which consequently led to down regulation of COX-2 and matrix metalloproteinase expression. Likewise, Kim et al. (2008) reported the corresponding activity for the two novel glycosides, isoliquiritin **(92)** and isoliquiritigenin **(93)** (Figure 8) from *Glycyrrhiza uralensi*. Isoliquiritigenin **(92)** have shown more pronounced activity against NO then isoliquiritin **(93)** with additional PGE_2_ inhibitory activity. Moreover, it was also able to decrease LPS-induced expressions of iNOS and COX-2 at the protein and mRNA levels in a concentration-dependent manner. In another study sphondin **(94)** (Figure 8) a rare compound from *Heracleum laciniatum* was able to exhibit wide range of anti-inflammatory activities. It was observed that sphondin **(93)** was able to reduce the biosynthesis of PGE_2_ in a dose dependent manner via suppressing the COX-2 activity in IL-1α induced RAW macrophage cells. A similar study was conducted by Zhou et al. (2008) focusing anti-inflammatory activity of 4-Methoxyhonokol **(95)** (Figure 8) isolated from *Magnolia obovata*. Results clearly suggest that 4-Methoxyhonokol **(95)** potentially inhibited the production and release of NO and PGE_2_ via mediating the activity gene expression of COX-2 and iNOS mRNA. In addition 4-Methoxyhonokol **(95)** blocked the NF-κB and MAPKs activation in LPS-stimulated RAW264.7 cells. Similar activity was reported for another lignin, schisandrin **(96)** (Figure 8) isolated from *Schisandra chinensis*. Schisandrin **(96)** significantly inhibited production of NO and PGE_2_ and gene expression of COX-2 and iNOS by suppressing the NF-κB, JNK, and p38 MAPK activation in RAW macrophage cell. In another phytochemical analysis carried out on *Boerhaavia diffusa* afforded 5 new and 4 known rotenoids. Among all the isolated compound boeravinone B **(97)** (Figure 8) have exhibited most significant COX1 and COX-2 activity with an IC_50_ value of 21.7 ± 0.5 and 25.5 ± 0.6 μM. Likewise in a similar study macrolide archazolid A (ArcA) **(**98**)** (Figure 8) from the *myxobacterium Archangium gephyra* was tested against LOX-5 and mPGES-1 inhibitory activity to acces its anti-inflammatory activity. The results suggested that ArcA able to significantly inhibited the gene expression of LOX-5 and mPGES-1 in LPS induced human blood with an IC_50_ value of 11 μM ± 0.2 and 8 μM ± 0.2 log units respectively. Similar activity was reported in the study where naturally occurring acylphloroglucinol myrtucommulone (MC) (99) (Figure 8) from *Myrtus communis* L. (myrtle) was tested for its anti-inflammatory activity in IL-1β-stimulated A549 cells. The suggested that MC able to significantly inhibited the mPGES-1-mediated conversion of PGH_2_ to PGE_2_ with an IC_50_ of 1 μM. However, in the same study MC failed to show any activity against COX-2 even at higher concentrations, which completely suggest that the fall in the PGE_2_ production observed in the current study is due to mPGES-1 gene suppression activity (Reker et al., 2014).

## Conclusion

Numerous classes of compounds have been explored in last two decades with significant anti-inflammatory activity. Flavonoid, terpinoids, alkaloids, and stilbenoids are the major class of compounds with potent COX-2 inhibitory activity. Although majority of flavonoids show more selectivity toward COX-1 isoenzymes. However, several studies have suggested that same compounds were significantly able to inhibit the COX-2 activity in *in-vivo* rate models, which suggest an alternative mechanism of action of COX-2 inhibition for flavonoids including kaempferol (47), myricetinglucuronide (49), and anthocyanin **(51)**. Alkaloids are very potent bioactive class of compounds with significant anti-inflammatory activity. Berberine **(1)** form *Berberis* sp. exhibited most significant COX-2 activity *in-vitro* and animal studies. Furthermore, the gene suppression activity of berberine imparts additional COX-2 suppression through inhibition of gene promoter proteins (AP-1, Mcl-1, and Akt). Hence making it the most suitable candidate for alternative therapeutic option for treating inflammation. However, few animal studies have indicated that at higher doses Berberine losses its COX-2 selectivity and may causes COX-1 associated gastric ulceration. Hence more toxicological studies need to be carried out in order to validate and standardize the therapeutic efficacy of berberine. Moreover, in the light of the above-mentioned studied capillarisin **(63)** and ginsenosides **(65)** have also shown potential to be serve as a potential therapeutic option due to their gene suppressing activity against MyD88/TIRAP, iNOS, and COX-2. More over both compounds can suppress the transcriptional activity of NF-κB, Akt, and MAPKs via blocking the LPS induced activation. Following are the list of the natural products with significant COX-2 and COX-2 mediated PGE_2_ inhibitory activity along with their IC_50_ values, berberine **(1)** 2.1 μM, rutaecarpine **(2)** 0.28 μM, 16aH,17-iso-valerate-ent-kauran-19-oic acid **(9)** 1.1 μM, ent-kaur-16-en-19-oic acid **(10)** 1.2 μM, ent-pimara-8(14), 15-dien-19-oic acid **(11)** 1.5 μM, arteminolide B **(12)** 7.17 μM, fomitopinic acid A **(14)** 0.15 μM, fomitoside E **(15)** 1.01 μM, fomitoside F **(16)** 1.15 μM, cyclomargenyl-3-O-β-caffeoyl ester **(21)** 10 μM, curdione **(24)** 1.1 μM, koetjapic acid **(27)** 1.05 μM, 3-oxoolean-12-en-30-oic **(28)** 1.54 μM, and betulinic acid **(29)** 2.59 μM, 7-angeloyl-12-acetyl-8-methoxyindol **(30)** 0.003 μM, aiphanol **(32)** 9.9 μM and isorhapontigenin **(33)** 6.2 μM, (+)-catechin **(39)** 3.3 μM, aciculatin **(46)**, myricetinglucuronide **(49)** 2.4 μM, taiwanin **C (80)** 0.12 μM. Moreover, all the above stated compounds can be future therapeutic alternative for treating inflammation associated diseases including neurodegenerative diseases, rheumatisms, and various cancers, where excessive COX-2 activity and PGE_2_ production plays significant role in development and progression.

## Author contributions

All authors listed have made a substantial, direct and intellectual contribution to the work, and approved it for publication.

### Conflict of interest statement

The authors declare that the research was conducted in the absence of any commercial or financial relationships that could be construed as a potential conflict of interest.
